# A Novel Fluorescent Dye Invades Mitochondria to Selectively Kill Cancer Stem Cells via Increased ROS Production

This article has been retracted.

**DOI:** 10.1155/2021/4763944

**Published:** 2021-10-13

**Authors:** Bei-Bei Zhang, Jun-gang Liu, Xian-Yu Bai, Yuan-Jiao Huang, Ning Xu, Tao Ren

**Affiliations:** ^1^Institute of Biomedical Research, Yunnan University, Kunming, China; ^2^Guangxi Medical University Affiliated Cancer Hospital, Nanning, China; ^3^Graduate School, Guangxi Medical University, Nanning, China; ^4^Life Science Institute, Guangxi Medical University, Nanning, China; ^5^School of Basic Medical Sciences, Guangxi Medical University, Nanning, China; ^6^The Fifth Affiliated Hospital of Guangxi Medical University, Nanning, China

## Abstract

Development of multiple agents has a significant impact on the cancer diagnosis and therapy. Several fluorescent dyes including near-infrared (NIR) fluorescent agents have been already well studied in the field of photodynamic therapy (PDT). In the present study, we reported a novel fluorescent dye could obviously inhibit cancer cell proliferation with slight toxic effects on the biological organism. Furthermore, it displayed selective staining on cancer cells, particularly on cancer stem cells (CSCs), rather than normal cells. Mechanically, this dye preferred to invading mitochondria of cancer cells and inducing overwhelming reactive oxygen species (ROS) production. The *in vivo* experiments further demonstrated that this dye could image cancer cells and even CSCs in a short-time intratumor injection manner using a zebrafish model and subsequently inhibit cancer cell proliferation after a relatively long-time drug exposure. Taken together, the future development of this agent will promise to make an essential contribution to the cancer diagnosis and therapeutics.

## 1. Introduction

Cancer is a heterogeneous disease and a major cause of death in the world. Cancer stem cell (CSC) theory presents that cancer is a stem cell disease, and CSCs are characterized by the drug resistance as well as the cancer recurrence [1, 2]. As the Achilles' heel against cancer, more and more therapeutic strategies are developed to eradicate CSCs. Many studies focus on CSC biology to unravel the mechanism and discover novel therapeutic targets or develop anti-CSC drugs [3, 4]. Two decades ago, leukemia stem cells (LSCs) in chronic myeloid leukemia (CML) were firstly discovered and characterized in the field of CSCs [5]. LSCs show a malignant seed of the disease, which is believed to induce drug resistance and relapse [6]. Although several target therapies including imatinib, a BCR-ABL tyrosine kinase inhibitor, have revolutionized the CML therapy as a classic model for targeted therapy in other cancer types, their efficacies against CSCs have been challenged [7, 8]. Recently, some novel rationales have been determined for the investigation of novel drug development including combination therapy and development of novel directions via targeting mitochondrial metabolism to eradicate therapy resistance [9, 10].

Numerous different clinical drugs or preclinical compounds are used for imaging cancer and even simultaneously present anticancer effects. Particularly, several near-infrared (NIR) dyes have shown well *in vivo* cancer imaging and cancer killing effects [11–13]. Researchers have already even tried to apply them in the precision oncotherapy [14, 15]. Several cyanine dyes or nanomicelles were used for mitochondria fluorescence imaging in cancer and highly efficient fluorescence imaging-guided photothermal therapy (PTT) [16–18]. In addition, several other fluorescent compounds even suggest their potentials as novel anti-CSC agents [19, 20]. For these fluorescent dyes, simultaneous cancer targeting, imaging, and cancer killing are a major advantage for cancer biology research and are expected to contribute to the future cancer therapy directions including photodynamic therapy (PDT) [21–23]. Furthermore, several specific membrane molecules targeting cancer cells have already been used in the *in vivo* NIR photoimmunotherapy field [24].

Zebrafish is the next-generation model organism. This species has the advantages of simple breeding, low price, *in vitro* fertilization, strong reproductive ability, short sexual maturity cycle, transparent embryos, and 87% similarity to human genes [25]. The development process and disease process are very similar to human development as well as the occurrence and development of human diseases [25]. At present, there are thousands of human disease-zebrafish models. In the field of cancer research and anticancer drug screening, a variety of transplantation, induction, and transgenic models are established in zebrafish, which can be used not only to study the effects of compounds on cancer cell proliferation and metastasis but also explore the mechanism of tumor angiogenesis and even evaluate the potential cardiotoxicity of anticancer drugs [8, 26, 27].

In the present study, we reported a novel fluorescent dye could obviously inhibit CSC proliferation *in vitro* and *in vivo* with slight toxic effects on the biological organism. Mechanically, this dye preferred to invading mitochondria of cancer cells and inducing overwhelming ROS production. Taken together, the future development of this agent will promise to make essential contribution to the diagnosis and therapeutics of the cancer disease.

## 2. Materials and Methods

### 2.1. Cell Proliferation Assay

K562 cells and the cells stable transfected with the Kusabira-Orange (KOr) fluorescent protein or blue fluorescent protein (BFP) were, respectively, cultured in the basic RPMI-1640 medium (Gibco) supplemented with 10% heat-inactivated FBS (Life Technologies), 100 U penicillin G/ml, and 100 *µ*g streptomycin/ml (Sigma-Aldrich) at 37°C in 5% CO_2_. The cell proliferation assay was performed using the CellTiter-Glo luminescent cell viability assay kit (Promega, Madison, WI, USA) according to the manufacturer's instructions.

### 2.2. ALDH-Positive Putative CSC Preparation

Aldehyde dehydrogenase (ALDH) positive and negative cells were sorted using an ALDEFLUOR assay kit (STEMCELL Technologies, Vancouver, Canada) followed by FACSAria flow cytometry (BD Biosciences) according to the manufacturer's instructions.

### 2.3. Mitochondria Staining

Cell and organelle were observed by immunofluorescence staining and confocal microscopy. As for the mitochondria staining in the alive cells, the MitoTracker™ Green dye (Thermo Fisher, Waltham, USA) was used according to the manufacturer's instructions.

### 2.4. ROS Measurement

The intracellular ROS level was measured using the CellROX detection reagent (Thermo Fisher, Waltham, USA). Hoechst 33342 dye was used for the nucleus staining. The images were captured using the ImageXpress Micro high-content screening system (Molecular Devices, Sunnyvale, USA). Cell fluorescence was quantified using the accompanying MetaXpress software (Molecular Devices, Sunnyvale, USA).

### 2.5. Cancer Mass *In Vivo* Imaging and Evaluation

The ALDH-positive and negative cell population of K562 cells were injected into the yolk sac of the transparent 48-hpf (hpf, hour postfertilization) zebrafish line (Tg: fli-EGFP) as described in the previous studies [8, 28]. The xenografted zebrafish were subsequently maintained at 32°C, and the successful cancer xenograft models with visible cancer mass were collected on the next day (1 dpi, day postinjection). As for short-time cancer imaging, the fluorescent dye was injected into the tumor mass and obtained images after 1 h; as for the anticancer effect evaluation, the cancer xenograft models were imaged on 1 dpi and exposed for 48 h to egg water containing the fluorescent agent and imaged again on 3 dpi. The cancer imaging and relative fluorescence intensity for each zebrafish were analyzed using an imaging-based method and MetaXpress software (Molecular Devices, Sunnyvale, USA). After the experiments, zebrafish used were sacrificed by an overdose of anesthesia.

### 2.6. Statistical Analysis

Data were shown as the mean ± SEM. The differences between two groups were analyzed using Student's *t*-test, and *P* value less than 0.05 was considered significantly different.

## 3. Results

### 3.1. A Novel Fluorescent Dye Obviously Inhibits Cancer Cell Proliferation with Slight Toxic Effects on the Biological Organism

To develop the novel biological chemicals, we tested a series of compounds and found one agent represented interesting biological characters. The chemical structure of one hit compound is shown in Figure 1(a). Interestingly, we first discovered that this compound could obviously inhibit the proliferation of BCR-ABL + CML K562 cells at 0.1 *μ*M, 0.33 *μ*M, and 1 *μ*M after 24 h exposure (*P* < 0.01, respectively; Figure 1(b)). Particularly, 1 *μ*M compound treatment has already killed more than 80% cancer cells. To determine the toxic side effects, we directly used 3 dpf (dpf, day postfertilization) zebrafish embryos as the model and found that as high as 20 *μ*M compound exposure for 48 h displayed nearly no effects on their survival ratios and morphology phenotypes, although we detected that the red fluorescent signal appeared in the whole fish body under the Cy5 microscopy filter and green fluorescent signal in the yolk sac under the GFP microscopy filter with a currently unknown reason (Figure 1(c)). There is no fluorescent signal detected under other available filters. Taken together, these data suggest that this novel fluorescent dye could be detected under the Cy5 filter and obviously inhibit leukemia cell proliferation with slight toxic effects on the biological organism.

### 3.2. Effects of the Staining on Cancer Cells, Particularly on CSCs *In Vitro*

To further explore the cancer selectivity of this agent, we collected the zebrafish blood cells as the model of normal cells, although these cells display smaller size than K562 leukemia cells. Interestingly, we found that 5 *μ*M compound exposure for 15 min could not obviously stain these normal blood cells, but the compound showed obvious staining on the K562-KOr cells under the same condition (Figure 2(a)). Statistically, the K562-KOr cells represented much higher integrated fluorescent intensity than the normal blood cells after this agent exposure (*P* < 0.01, Figure 2(b)). These data suggested that this novel agent preferred to staining cancer cells than normal cells and somehow explained that why there were slight toxic effects on the biological organism but kill cancer cells. Moreover, previous research has proved that ALDH(+) cells could be deemed as the putative leukemia stem cells [29]. Importantly, in the present study, we discovered that ALDH(+) cells showed higher integrated fluorescent intensity than the ALDH(−) cells (*P* < 0.01, Figures 2(c) and 2(d)). Clearly, these data indicated that this novel fluorescent dye preferred to staining on cancer cells, particularly on CSCs.

### 3.3. Targeting Mitochondria of Cancer Cells as the Main Intracellular Dye Accumulation Site

Since we discovered that the cancer cells were selectively stained by this compound, next we wonder the exact subcellular localization. To label the organelle, we used the MitoTracker Green fluorescent dye to stain mitochondria (green signal) and found that most of the novel fluorescent dye staining (red signal) could colocalize well with the green signal (Figure 3(a)) in K562 leukemia cells. The integrated density also showed consistent values in different image areas (*X*-distances) (Figure 3(b)). Clearly, the data suggested that this novel fluorescent dye mainly targeted mitochondria of cancer cells as the intracellular dye accumulation site.

### 3.4. Effects on the ROS Level in CSCs

These above data uncovered that this novel fluorescent dye preferred to gathering into mitochondria in cancer cells, especially in CSCs. Since we have already detected that the mitochondria of cancer cells were the main intracellular accumulation site of this novel compound, next we would measure the reactive oxygen species (ROS) level in ALDH(+) cells because mitochondria in cancer cells were characterized as the main source of ROS overproduction, which played an important role in CSC biology [30, 31]. Interestingly, we found that the compound treatment could obviously increase the intracellular ROS level in these ALDH(+) cells (Figures 4(a) and 4(b)). Taken together, these data indicated that the dye accumulated in mitochondria might stimulate the CSCs to produce overwhelming ROS, which might be one reason for their anticancer effects.

### 3.5. Effects of the Staining on Cancer Cells, Particularly on CSCs *In Vivo*

Since we have known that this novel fluorescent dye could image and kill cancer cells *in vitro* from above experiments already performed, we next wonder the *in vivo* effects of this fluorescent dye. We first sorted ALDH(+) and ALDH(−) K562-BFP cells and then injected them into the zebrafish embryos, respectively. On the next day, we collected the successful xenograft on 1 dpi (dpi, day postinjection) and subsequently injected the fluorescent dye into the tumor mass and obtained the images after 1 h. Clearly, the fluorescent dye nearly labels the whole cancer mass for both ALDH(+) and ALDH(−) cells, respectively (Figure 5). The results suggested that this fluorescent dye could also stain on cancer cells, particularly on CSCs *in vivo*.

### 3.6. The Novel Fluorescent Dye Inhibits CSCs *In Vivo*

Since this fluorescent dye could stain on CSCs *in vivo*, we next constructed the ALDH(+) K562-KOr cell xenografted zebrafish. Similarly, the successful xenografts on 1 dpi were selected and imaged. Subsequently, we put these embryos in egg water containing this novel fluorescent dye for 48 h and imaged these xenografts on 3 dpi again in a 96-well plate. The cancer cell mass was analyzed and quantified before and after this dye exposure for each xenografted zebrafish (Figure 6(a)). Statistically, this novel fluorescent dye could inhibit CSCs *in vivo* indicated by these above experiments (*P* < 0.01, Figure 6(b)). Taken together, the results suggested that this fluorescent dye could also inhibit CSCs *in vivo*.

## 4. Discussion

Organic dyes have been applied in biology and medical research for many years. For three decades, the mitochondrial probe rhodamine 123 and its analogs have been adapted for testing the viability of pulsating myocardial cells [32]. As the representative fluorescent contrast agents, polymethine cyanine dyes such as IR-786 and indocyanine green (ICG) have also long been used in clinical and experimental NIR imaging [33–35]. Moreover, a NIR heptamethine cyanine dye named IR-780 iodide showed preferential accumulation in many tumor cells and represented biocompatible properties for the imaging of the sentinel lymph node [36, 37]. Here, we reported a novel fluorescent dye also showed preferential cancer cell, especially CSC, accumulation compared with normal cells. Similarly, this dye also represented cancer imaging and cancer inhibition by invading mitochondria and inducing overwhelming ROS (Figure 7). These characters make it an attractive leading compound for the diagnosis and therapeutics of future cancer imaging and therapy.

Mitochondria are important organelles. They provide energy to sustain the metabolic needs of the cells, particularly the cancer cells. Moreover, they also provide building blocks for the new cells, especially for the rapid proliferated cancer cells, and control the redox homeostasis, oncogenic signaling pathway, immunity interaction, and apoptosis [38]. There is no doubt that mitochondria act a central role and play multiple functions in the cancer progression. Therefore, targeting mitochondria in cancer has become the novel concept and approach in the war against cancer, which provides many therapeutic opportunities including immunotherapy [39]. In the current study, we found that the fluorescent dye accumulated in mitochondria; the reason might be that there was a relatively higher mitochondrial membrane potential in cancer cells than that of normal cells [40]. Most lipophilic cationic dyes were proved to selectively target the mitochondria of cancer cells due to the higher negative inside transmembrane potentials of the mitochondria [41, 42]. Lipophilic cations preferentially accumulate in the cells with higher mitochondrial membrane potential [43]. The CSCs might have higher membrane potential than other cell populations, which induced the most dye accumulation [31]. The view was supported by one previous study in that the CSC biomarker CD133 was expressed in these higher mitochondrial membrane potential cells, but not in the other cells [44].

The main prominent source of intracellular ROS is from mitochondria. ROS are closely related with cancer development, including every stage of the initiation, promotion, and progression [45]. ROS overproduction is one hallmark of cancer cells. It is well known that ROS plays multiple roles in inducing genomic instability, modifying the gene expression, and participating in signaling pathways [30]. In the current study, we observed that this dye mainly accumulated in the mitochondria, which might damage the respiratory electron-transport chain and produce the stimulus to trigger the overwhelming ROS production in mitochondria. There is a crosstalk between the ROS, mitochondria, and nucleus. Obviously, the ROS level and resistance ability in niches of CSCs are also different due to their characters. Similar to our finding about this novel fluorescent dye, a lot of (pre-) clinical anticancer drugs targeting different species of ROS have been developed [45, 46]. Some novel anti-CSC therapeutic approaches are also reported to be related with the modulation of redox signaling pathways [47, 48].

Cancer stem cells (CSCs) are the initiators of cancer occurrence, development, and recurrence. In the present study, ALDH(+) cells were deemed as the model of putative CSCs because previous studies have proved that cell populations with high ALDH activity exhibit CSC properties [49, 50]. The ALDH(+) K562 cell population expressed the CSC markers CD133 and CD34 and showed higher tumorigenesis and imatinib resistance than ALDH(−) cells in earlier studies [8, 51–53]. Targeting this unique population of cancer cells would provide a novel rationale. The therapeutic agents often represent less toxicity than regular chemotherapeutic drugs, which often kill bulk cancer cells and normal cells, but are impotent for CSC killing. The elevated ROS levels might trigger the differentiation of CSCs including LSCs, and overwhelming concentration of ROS mainly produced from mitochondria may be an optimal treatment to eradicate this cell population during cancer therapy [54, 55].

## 5. Conclusion

Taken together, in the present study, we found one novel fluorescent dye could obviously image and inhibit cancer cells including CSCs via invading mitochondria and inducing overwhelming ROS production. The future development of this anticancer reagent characterized by slight side effects will provide an alternative strategy for cancer diagnosis and therapy.

## Figures and Tables

**Figure 1:** A novel fluorescent compound selectively inhibits cancer cell proliferation. (a) The chemical structure of the discovered novel fluorescent dye. (b) Cell proliferation status of K562 cells treated with the compound for 24 h in different concentrations; ^*∗∗*^*P* < 0.01 and *n* = 3. (c) Morphology phenotype of the 5 dpf (dpf, day postfertilization) zebrafish embryos observed under different (bright field, GFP filter, and Cy5 filter) microscopy filters after treatment with the compound in different concentrations from 3 dpf for 48 h. There is no fluorescent signal detected under other available microscopy filters.

**Figure 2:** Selective staining on cancer cells, particularly on CSCs. (a) Representative images of zebrafish blood cells and K562-KOr cancer cells stained for 15 min in 5 *μ*M compound exposure; blue: nucleus staining by Hoechst 33342; green: KOr expressed yellow fluorescence merged with the blue nucleus; red: the compound displayed red fluorescence. (b) Integrated fluorescence intensity of the compound staining on zebrafish blood cells and K562-KOr cancer cells. (c) ALDH(−) and ALDH(+) cells of K562 cells were stained for 24 h in 1 *μ*M compound exposure; blue: Hoechst 33342 for nucleus staining; red: the compound displayed red fluorescence. (d) Integrated fluorescence intensity of the compound staining on K562 ALDH(−) and ALDH(+) cells.

**Figure 3:** Mitochondria staining in the cancer cells. (a) Confocal images of K562 cells stained using 5 *μ*M compound (red) for 40 min and 400 nM MitoTracker Green dye for 15 min. (b) Quantification of the red and green signals for one virtual line set along the *X*-axis direction in the middle of the *Y*-axis direction.

**Figure 4:** ROS production in the K562 ALDH(+) cells. (a) Representative images of the ROS status in K562 ALDH(+) cancer cells with or without 1 *μ*M compound exposure for 24 h. (b) Integrated fluorescence intensity of the ROS signals in K562 ALDH(+) cancer cells with or without 1 *μ*M compound exposure for 24 h.

**Figure 5:** Selective staining on cancer cells *in vivo*. Representative images of the ALDH(−) and ALDH(+) K562-BFP zebrafish xenograft (1 dpi; dpi, day postinjection) after 10 *μ*M compound intratumor injection for 1 h.

**Figure 6:** Selective inhibition of CSCs *in vivo*. (a) Representative images of the ALDH(+) K562-KOr cell zebrafish xenograft (1 dpi and 3 dpi; dpi, day postinjection) before and after 1 *μ*M compound exposure for 48 h. (b) Quantification of ALDH(+) K562-KOr cells in the zebrafish xenograft (3 dpi normalized to 1 dpi) about the anticancer effects of 1 *μ*M compound exposure for 48 h. ^*∗*^*P* < 0.05 and *n* = 4.

**Figure 7:** A working model for the application of the fluorescent dye in cancer.

## Data Availability

The datasets used and/or analyzed during the current study are available from the corresponding author upon reasonable request.

## Abbreviations

NIR: Near-infrared
PDT: Photodynamic therapy
CSC: Cancer stem cell
ROS: Reactive oxygen species
LSC: Leukemia stem cell
CML: Chronic myeloid leukemia
PTT: Photothermal therapy
KOr: Kusabira-Orange
BFP: Blue fluorescent protein
ALDH: Aldehyde dehydrogenase
hpf: Hour postfertilization
dpf: Day postfertilization
dpi: Day postinjection
ICG: Indocyanine green.
